The article "Green Synthesis of Metallic Nanoparticles and Their Potential Applications to Treat Cancer" was retracted in 2023. Reason: plagiarized images.

# Green Synthesis of Metallic Nanoparticles and Their Potential Applications to Treat Cancer

**DOI:** 10.3389/fchem.2020.00799

**Published:** 2020-10-29

**Authors:** Dan Zhang, Xin-lei Ma, Yan Gu, He Huang, Guang-wei Zhang

**Affiliations:** Department of Cardiology, First Hospital of Jilin University, Changchun, China

**Keywords:** metallic nanoparticles, green synthesis, extracellular, intracellular, tissue engineering, bio-detection

## Abstract

Nanoparticle synthesis using microorganisms and plants by green synthesis technology is biologically safe, cost-effective, and environment-friendly. Plants and microorganisms have established the power to devour and accumulate inorganic metal ions from their neighboring niche. The biological entities are known to synthesize nanoparticles both extra and intracellularly. The capability of a living system to utilize its intrinsic organic chemistry processes in remodeling inorganic metal ions into nanoparticles has opened up an undiscovered area of biochemical analysis. Nanotechnology in conjunction with biology gives rise to an advanced area of nanobiotechnology that involves living entities of both prokaryotic and eukaryotic origin, such as algae, cyanobacteria, actinomycetes, bacteria, viruses, yeasts, fungi, and plants. Every biological system varies in its capabilities to supply metallic nanoparticles. However, not all biological organisms can produce nanoparticles due to their enzymatic activities and intrinsic metabolic processes. Therefore, biological entities or their extracts are used for the green synthesis of metallic nanoparticles through bio-reduction of metallic particles leading to the synthesis of nanoparticles. These biosynthesized metallic nanoparticles have a range of unlimited pharmaceutical applications including delivery of drugs or genes, detection of pathogens or proteins, and tissue engineering. The effective delivery of drugs and tissue engineering through the use of nanotechnology exhibited vital contributions in translational research related to the pharmaceutical products and their applications. Collectively, this review covers the green synthesis of nanoparticles by using various biological systems as well as their applications.

## Introduction

Nanotechnology is amongst the most widely used technologies in translational research. The development of metallic nanoparticles employing biological materials by an eco-friendly approach has attracted significant attention. Nanotechnology deals with particles of a size ranging from 1 to 100 nm, their synthesis strategy, and manipulation. This knowledge domain naturally commingles all the fields of natural sciences together with chemistry, physics, biological sciences, engineering, materials science, and computational sciences for the formulation of nanostructures (Shenton et al., 1999; Medvedeva et al., 2007). The nanostructures have different applications attributable to their new or increased properties (Tang et al., 2007; Thakkar et al., 2009) depending upon their size, distribution, and morphology. It has applications in various fields including biomedical, catalysis, chemical industries, cosmetics, drug delivery, electronics, environment, energy science, food and feed, health care, mechanics, optics, space industries, non-linear optical devices, single-electron transistors, and photo-electrochemical applications. The metallic nanoparticles are considered one of the most promising systems for all the aforementioned functions (Wang et al., 2005; You et al., 2013; Singh et al., 2016).

The article "Green Synthesis of Metallic Nanoparticles and Their Potential Applications to Treat Cancer" was retracted in 2023. Reason: plagiarized images.

A nanoscale drug carrier acts as a single unit with respect to its properties and transport. These nanoclusters have narrow size distribution and a minimum of one dimension between 1 and 10 nanometers. The agglomerates of ultrafine particles, nanoclusters or nanoparticles, are nanopowders whereas nanocrystals are the crystals of nanoparticle size

There are two general strategies for the synthesis of nanomaterials: the top-down approach, wherein a larger structure is broken down into smaller pieces using chemical, physical, and biological energy; and the bottom-up approach, in which material is synthesized from the atomic level using various chemical, physical, or biological reactions to make a large nanostructure (Das et al., 2017). The chemical and biological methods are primarily accustomed to build nanostructured carriers (NC) employing this approach (Figure 1).

**Figure 1:** **(A,B)** Approaches and method of synthesis of nanoparticles.

The physical and chemical strategies are in-use for the synthesis of nanoparticles. The utilization of toxic chemicals could exert potential hazards like carcinogenicity, toxicity, and environmental toxicity (Gupta and Xie, 2018). The toxicity problems are quite prominent due to the use of hazardous substances such as reducing agents, organic solvents, and stabilizers. These chemicals prevent the agglomeration of colloids. The use of toxic solvents and chemical contaminations limits the use of nanoparticles in various clinical and biomedical applications (Hua et al., 2018). Therefore, a reliable, clean, biologically appropriate, and environmental-friendly techniques is indeed required to synthesize nanoparticles (Jain et al., 2010; Thakkar et al., 2010; Kulkarni and Muddapur, 2014). The biological synthesis of nanoparticles may prove to be an attractive alternative. It includes adoption of multicellular and unicellular biological entities- bacteria (Roh et al., 2001; Nair and Thalappil, 2002; Lengke et al., 2006; Husseiny et al., 2007; Joglekar et al., 2011), actinomycetes (Ahmad et al., 2003a,b; Sastry et al., 2005), fungi Mukherjee et al., 2001, 2002; Ahmad et al., 2002, 2005; Bhainsa and D'Souza, 2006, plants Philip, 2010; Kumar et al., 2011, viruses (Lee et al., 2002; Merzlyak and Lee, 2006; Khan et al., 2013), and yeasts (Dameron et al., 1989; Kowshik et al., 2003; Gericke and Pinches, 2006a,b). The biologically synthesized nanoparticles have a broad area to study with respect to their shape, size, composition, and physicochemical properties (Mohanpuria et al., 2008). Further, biological entities may operate as a pattern for the assembly, synthesis, and organization of the nanometer scale. The present review covers the use of biological routes for the synthesis of metal oxide and metal nanoparticles, and various factors affecting their synthesis, and possible mechanisms employed along with likely applications of nanoparticles formed using biological factories.

The article "Green Synthesis of Metallic Nanoparticles and Their Potential Applications to Treat Cancer" was retracted in 2023. Reason: plagiarized images.

## Biological Synthesis of Nanoparticles

Organisms have advanced to endure in environments of high concentrations of metals (Bisen et al., 1987, 1996; Khare and Bisen, 1991). These organisms may alter the chemical nature of the toxic metals by lowering their toxicity or making them non-toxic (Singh et al., 1989, 1993; Sharma and Bisen, 1992; Sharma et al., 2001). The formation of nanoparticles is the “consequence” of the resistance mechanism of an organism in contrast to a specific metal (Figure 2). The synthesis of “Natural” biogenic metallic nanoparticle synthesis is split into two categories:

**Figure 2:** Various biological synthesis of nanoparticles.

(a) **Bioreduction**: More stable forms of metal ions may be achieved by chemical reduction using biological means and is achieved by dissimilatory metal reduction. The metal ion is reduced and the enzyme is oxidized (Deplanche et al., 2010). This concludes in the production of impotent metallic nanoparticles which may be harmlessly recovered from a contaminated sample.

(b) **Biosorption**: The metal ions bind to the organism itself from an aqueous sample or soil sample. Either the metal ions are bonded to the cell wall or peptides are synthesized by some plants, bacteria, and fungi, and these synthesized peptides assembles into stable nanoparticulate structures (Yong et al., 2002).

The selection of biological methods for synthesis and engineering of nanoparticles is dependent upon several variables. The form of the metal nanoparticle to be synthesized is the most important variable. Resistance developed against a small number of metals by the organisms limit the choice of organisms. Following are a number of the microbial resources (algae, fungi, bacteria, viruses, and yeast) used for most of the frequently studied metal and metal salts nanoparticles consisting of copper, silver, gold, cadmium, platinum, palladium, cadmium sulfide, titanium dioxide, and zinc oxide (Mousavi et al., 2018; Gahlawat and Roy Choudhury, 2019).

The article "Green Synthesis of Metallic Nanoparticles and Their Potential Applications to Treat Cancer" was retracted in 2023. Reason: plagiarized images.

### Bacteria Mediated Synthesis of Nanoparticles

Pure gold nanoparticles were synthesized by bacterium, *Delftia acidovorans* (Johnston et al., 2013). Delftibactin is a small non-ribosomal peptide and is considered liable for the synthesis of gold nanoparticles as it is known to induce resistance against toxic gold ions. The transition metal, gold, did not exert toxicity toward bacterium due to the formation of inert gold nanoparticles (AuNPs) bound to delftibactin (Pantidos and Horsfall, 2014). A substitutive method for gold nanoparticle synthesis by the bacterium *Rhodopseudomonas capsulata* was shown to produce extracellular gold nanoparticles ranging in size from 10 to 20 nm via NADH-Dependant Reductase (He et al., 2007). Green products may act as a stabilizing and reducing agent for AuNPs synthesis and these preparations exhibit medicinal applications (Lee et al., 2020).

Palladium (Pd), one of the members of the Platinum Group Metals (PGM) has a compilation of highly catalytically active metals, and is being employed as a catalyst for hydrogenation and dehalogenation reactions. The heavy contamination of those bacteria that had been isolated from Alpine sites with that of heavy metals led to the synthesis of zero-valent Palladium (Pd^0^) nanoparticles (Schlüter et al., 2014). Amongst various bacteria isolated from the site, only Pseudomonas cells exhibited the potential to produce catalytically active Pd nanoparticles. Furthermore, they were able to carry out the reductive dehalogenation of congeners like tri and tetra-chlorinated dioxin. *Escherichia coli* synthesized Pd^0^ nanoparticles using hydrogenases present in the cells (Lloyd et al., 1998). Pd nanoparticles were synthesized on the bacterial cell envelope and may be separated easily.

The bacterium, *Bacillus licheniform*, reportedly produced silver nanoparticles (AgNPs) intracellularly (Kalimuthu et al., 2008). The production/synthesis of nanoparticles required 24 h and was demonstrated by the color modification of culture into dark brown after the augmentation of silver ions. However, as the nanoparticles were synthesized intracellularly an additional extraction step was required. Intracellular AgNPs were synthesized by the members of the *Bacillus* spp. subcultured in AgNO_3_ containing media and the reaction was completed in 7 days (Pugazhenthiran et al., 2009). The culture supernatant was tested for its capability to form metallic nanoparticles (Shahverdi et al., 2007) in 5 min. The extracellular production of nanoparticles is recommended compared to the intracellular synthesis due to the simple purification process with the increased production rate (Das et al., 2014).

The article "Green Synthesis of Metallic Nanoparticles and Their Potential Applications to Treat Cancer" was retracted in 2023. Reason: plagiarized images.

Green synthesis of AgNPs using lactic acid bacteria was demonstrated by Sintubin et al. (2009). *Lactobacillus* spp., *Pediococcus pentosaceus, Enterococcus faecium*, and *Lactococcus garvieae* was shown to synthesize the nanoparticles by many bacteria. The procedure of AgNP formation was proposed to be a two-step method. The biosorption of Ag ions on the cell wall was followed by a reduction of these ions resulting in AgNPs formation (Sintubin et al., 2009). Additionally, the cell wall could be thought to be a capping agent, maintaining their stability by stopping their aggregation.

The biosynthesis of Ag and AuNPs has been a focal point of research because of their antimicrobial attributes. The extensive studies were conducted to synthesize the metallic nanoparticles using Bacillus species due to their metal accumulating abilities (Pollmann et al., 2006; Kalimuthu et al., 2008; Pugazhenthiran et al., 2009). *Bacillus sphaericus* JG-A12 can collect excessive concentrations of Al, Cd, Cu, Pb, and U (Figure 3). The Uranium bioremediation from the aqueous environment was attributed to the S-layer proteins of *B. sphaericus*. It is a porous layer surrounding the bacterial cell and is made up of identical proteins, ~5–15 nm thick, with the pores ranging in size from 2 to 6 nm. The S-layer contributes up to 15% of the total proteins of the cell. The S-layer has been stated to be liable for the binding of heavy metals from the aqueous environments (Pollmann et al., 2006) with a capability to bind up to 20 mg U/g of protein, and the U binds to the phosphate and carboxyl and groups of the S-layer protein (Pollmann et al., 2006).

**Figure 3:** Green synthesis of nanoparticles by plants.

Copper (Cu) is not reportedly stable and is oxidized rapidly to copper oxide (CuO) (Baco-Carles et al., 2011). Therefore, Cu nanoparticles need to be stabilized as soon as they are formulated. The synthesis of Cu nanoparticles using *Morganella morganii* is proved with the help of intracellular uptake of Cu ions accompanied by the means of binding of ions to a metallic ion reductase or a comparable protein ensuring in the reduction of the ion to metallic Cu^0^ (Baco-Carles et al., 2011). The metallic Cu nanoparticles then accumulate extracellularly since they are effluxed out of the cell. *Morganella* sp. additionally extracellularly synthesized AgNPs (Parikh et al., 2008). The Cu nanoparticles synthesis using *M. morganii* may be due to an Ag resistance mechanism to provide elemental Cu nanoparticles through silE homolog to copper-binding protein from different microorganisms (Ramanathan et al., 2013).

The article "Green Synthesis of Metallic Nanoparticles and Their Potential Applications to Treat Cancer" was retracted in 2023. Reason: plagiarized images.

### Nanoparticle Synthesis Using Fungi

The production of AgNPs using fungi has been the focal point of investigation because of their applications in numerous industries such as antimicrobials and electronics (Rai et al., 2008; Ummartyotin et al., 2012). The capability of the fungus *Fusarium oxysporum* to synthesize AgNPs has been verified with sizes ranging from 5 to 15 nm which had been capped through fungal proteins to lead them to becoming stable. *Fusarium oxysporum* could also synthesize nanoparticles extracellularly (Rai et al., 2008; Ummartyotin et al., 2012) as compared to earlier studies in which intracellular production of Ag and AuNPs, lead sulfide (PbS), cadmium sulfide (Cds), molybdenum sulfide (MoS), and zinc sulfide (ZnS) nanoparticles intracellular production of Ag and AuNPs, cadmium sulfide (Cds), lead sulfide (PbS), zinc sulfide (ZnS), and molybdenum sulfide (MoS) had been reported (Ahmad et al., 2002, 2003a).

*Aspergillus fumigatus* is used to synthesize extracellular silver nanoparticles of larger sizes ranging from 5 to 25 nm as compared to *Fusarium oxysporum*, with the disadvantage of difficulty in anticipating the catalytic activity with the size difference in every batch (Bhainsa and D'Souza, 2006). However, the bio-production of AgNPs using *A. fumigatus* is an attractive prospect as organism reduces Ag ions into nanoparticles within 10 min of contact (Bhainsa and D'Souza, 2006). Fungus *Trichoderma reesei* could also be used for extracellular production of AgNPs with a size range of 5–50 nm nanoparticles. It took 72 h to synthesize AgNPs which was appreciably slower than *A. fumigatus* and *Fusarium oxysporum* (Ahmad et al., 2002, 2005; Bhainsa and D'Souza, 2006). Furthermore, the use of *T. reesei* has an advantage over the use of other fungi since it has been an extensively-studied organism which may be manipulated for the production of an excessive quantity of enzymes (Roy et al., 2008; Vahabi et al., 2011) and may help increase the rate of production of nanoparticles. However, the nanoparticles were not as homogenous as those which were produced by *A. Fumigates* (Bhainsa and D'Souza, 2006) and *F. oxysporum* (Ahmad et al., 2002). The fungal attribute to produce intracellular nanoparticles is helpful in getting rid of the fungus and its gathered metallic contaminant. A white-rot fungus (*Coriolus versicolor*) is suggested to provide and accumulate AgNPs extra and intracellularly by manipulating reaction conditions (Sanghi and Verma, 2008). Only a few fungi are considered to have the potential to synthesize gold nanoparticles despite the increasing demand in various fields. The small size of gold nanoparticles causes them to become more reactive and appropriate as compared to the bulk form to be used as precursors for electronics applications and catalysts (Mukherjee et al., 2001; Eustis and El-Sayed, 2006). The synthesis of AuNPs using *Verticillium* sp. by the biological reduction of AuCl_4_ localized on the surface of the mycelia (Mukherjee et al., 2001).

The article "Green Synthesis of Metallic Nanoparticles and Their Potential Applications to Treat Cancer" was retracted in 2023. Reason: plagiarized images.

Biological synthesis of Platinum nanoparticles (PtNPs) was carried out by the use of fungus *Neurospora crassa*. It produced single PtNPs (Platinum nanoparticles) intracellularly ranging in size from 4 to 35 nm in diameter. They may additionally synthesize spherical nano-agglomerates in the range of 20–110 nm diameter (Castro et al., 2013). Both biomass and extract of *N. crassa* were used to synthesize PtNPs. The PtNPs synthesized using the *N. Crassa* extract contains single-crystal nano agglomerates (Castro et al., 2011, 2013). PtNPs were also reportedly synthesized extra and intracellularly by *F. oxysporum* but with sub-optimal quantity when synthesized intracellularly (Riddin et al., 2006). The phytopathogenic fungus *F. oxysporum* and the endophytic fungus *Verticillium* sp. had been reported to synthesize magnetite (a common iron oxide) nanoparticles (MaNPs) intracellularly (Bharde et al., 2006).

The use of fungi for nanoparticles synthesis has some benefits over the use of bacteria namely; scaling up and easy downstream processing, the economic status, and an increased surface area provided by the fungal mycelia (Mukherjee et al., 2001). The higher amount of proteins secreted by using fungi should likely increase the productivity of nanoparticle synthesis but safety is compromised since a number of fungi are phytopathogenic and may pose a safety risk (Spadaro and Gullino, 2005). *Trichoderma asperellum* and *Trichoder mareesei* are non-pathogenic making them ideal for commercial applications (Nevalainen et al., 1994; Roy et al., 2008; Vahabi et al., 2011). *T. reesei* is broadly used in animal feed, food, paper, pharmaceuticals, and textile industries (Nevalainen et al., 1994).

### Nanoparticle Synthesis Using Yeast

Yeasts can absorb and accumulate a good quantity of lethal metals from their adjacent areas due to their large surfaces (Bhattacharya and Gupta, 2005; Mandal et al., 2006). Yeast uses a range of detoxification mechanisms to adapt to toxic metals such as bio-precipitation, chelation, extracellular sequestration and bio-sorption. These mechanisms adapted through yeast cells are used during nanoparticle synthesis to form and increase the durability of nanoparticles, giving rise to variation in particle size, particle properties, and location (Hulkoti and Taranath, 2014). The intracellular synthesis of CdS quantum dots turned into confirmed via *Candida glabrata* when exposed to cadmium salts (Dameron et al., 1989). The growth phase of yeast *Schizosaccharomyces pombe* cells and the formation of CdS quantum dots are linked together (Kowshik et al., 2002a,b). *Torulopsis* sp. synthesizes PbS quantum dots when exposed to Pb^2^ ions and *Pichia jadinii* synthesizes Au nanoparticles intracellularly. The size range of these nanoparticles is from a few nanometers to around 100 nm. The morphological characteristics of these nanoparticles were easily conducted by monitoring the cellular activities and growth of *P. jadinii* during the synthesis of the nanoparticle (Gericke and Pinches, 2006a,b). The use of metallic nanoparticles has become vital due to their safety and prospective applications.

The article "Green Synthesis of Metallic Nanoparticles and Their Potential Applications to Treat Cancer" was retracted in 2023. Reason: plagiarized images.

### Nanoparticles Synthesis Using Cyanobacteria (Blue Green Algae)

Green and valuable synthetic techniques have attracted great interest in the synthesis of nanoparticles (Sundrarajan and Gowri, 2011). Cyanobacteria strains are an inexpensive eco-friendly tool for nanometal formation. Cyanobacterial technology offers the merits of eco-friendly methods, such as timesaving for large-scale production at ambient temperatures. They grow much faster compared to the plants and could easily be manipulated as needed. Studies on molecular biology and ecology regarding synthesis of nanoparticles offer a great opportunity for efficient development of application-oriented nanoparticles. The common cyanobacterial strains used in nanoparticle biosynthesis vary from unicellular and colonial species. Colonies might form sheets, filamentous, or even hollow balls. They may fix atmospheric nitrogen besides fixing the atmospheric carbon dioxide during photosynthesis. Some strains grow in dark under organotrophic/chemotrophic/lithotrophic conditions offering a wide range of modes of nutrition with normal plants-like photosynthesis. Few strains exhibit symbiotic conditions with lichen (Fungi), bryophytes (Liverworts), gymnosperms (Cycas), and with higher plants (Macrozamia). They require a lesser quantity of chemicals as they are all photoautotrophic and may also grow under the chemo-autotrophic condition in light and dark.

Out of the 30 different strains of cyanobacteria (unicellular, colonial, undifferentiated and differentiated filamentous) studied for the silver nanoparticles biosynthesis, the filamentous heterocystous strain *Cylindrospermum stagnale* was the best organism synthesizing nanoparticles of 38–40 nm (Husain et al., 2015). In general, the time frame varied from 30 to 360 h, and the size varied from 38 to 88 nm (Husain et al., 2015). The techniques of synthesis of AgNPs using cyanobacteria *Spirulina platensis* and *Nostoclinckia* have been studied (Cepoi et al., 2014). There is a need to understand the optical conditions of the interaction among the biomass and solution containing Ag ions that may allow nanoparticles without biomass degradation at the time of Ag nanoparticle formation (Cepoi et al., 2014; Hamouda et al., 2019). The green synthesized silver nanoparticles via simple biological protocol using *Oscillatoria limnetica* aqueous extract that had provided both a decreasing and stabilizing agent for the biosynthesis of nanoparticles by suspending the live and washed biomass into the AgNO_3_ solution and by adding AgNO_3_ into a cell-free culture liquid (Patel et al., 2015) assessed the selected strains of cyanobacteria for the ability to synthesize AgNPs. Around 14 out of 16 tested strains have been utilized for the AgNPs biosynthesis. Mostly, AgNPs have been formed in the presence of biomass in addition to the cell-free culture media indicating that the Ag-NPs formation technique engages an extracellular compound inclusive of polysaccharide. TEM evaluation revealed that nanoparticles were set in an organic matrix. AgNPs varied in shape and sizes that ranged between 13 and 31 nm, depending upon the organism used (Patel et al., 2015). With the exception of one strain of Cyanobacterium *Limnothrix* sp., all strains confirmed the antibacterial activity of Ag-NPs (Patel et al., 2015). For the gold nanoparticles green synthesis, *Lyngbya majuscula* and *Spirulina subsalsa* were investigated as bioreagents. The cyanobacterial biomass turned purple within 72 h of incubation at 15 mg L-1 Au^3+^ solution, indicating an intracellular reduction of Au^3+^ to Au^0^ and subsequent formation of gold nanoparticles. *Spirulina subsalsa* showed the synthesis of spherical nanoparticles of ~5 to ~30 nm in diameter along with very few nanorods. *Lyngbya majuscule* showed the presence of spherical and hexagonal nanoparticles of ~2 to ~25 nm in diameter. The reduction of Au^3+^ to Au^0^ was proved by the XRD study. FTIR analysis indicated the presence of protein shells around the gold nanoparticles (Parial and Pal, 2011). The biosynthesis of AgNPs and their antimicrobial property and photocatalytic activity for photodegradation of organic dye were studied by San Keskin et al. (2016). The characterization of synthesized Ag nanoparticles was carried out by UV–Vis spectrophotometer (surface plasmon resonance band at 430–450 nm). The Attenuated Total Reflection Fourier Transform Infrared Spectroscopy (ATR-FTIR) study confirmed the reducing nature of proteins. The Scanning electron microscopy (SEM) and Transmission electron microscopy (TEM) were used to determine the structure of AgNPs and was found to be spherical. The AgNPs showed photocatalytic activity that is photodegradation of organic dye i.e., methylene blue. It was shown that methylene blue was degraded by ~18% within 4 h with biosynthesized AgNPs (San Keskin et al., 2016). The biosynthesis of AgNPs has been efficaciously performed with the use of bloom-forming filamentous undifferentiated cyanobacterium *Plectonema boryanum* which reacted with solution of AgNO_3_ (~560 mg/L Ag) for up to 28 days at 25–100°C. The precipitation of spherical AgNPs and octahedral silver platelets (of up to 200 nm) in solutions is promoted by interaction of cyanobacteria with AgNO_3_ Solution. The mechanism of formation of AgNPs via cyanobacteria may involve the metabolic processes in which nitrate is used at 25°C, and organics are released from the lifeless cyanobacteria at 25–100°C (Lengke et al., 2006, 2007). The cyanobacterium *Gloeocapsa* sp. was an effective strain for nanosilver production (Al-Katib et al., 2015). The extracellular synthesis of AgNPs was initially detected by visual inspection for color changing of the cultured flasks solutions from transparent to brown then black, as well as nanoparticles characterization through UV-Vis spectrophotometer and Fourier Transform Infrared spectroscopy (FTIR) with characteristic surface Plasmon absorption peaks at range 400–450 nm. The FTIR spectrum data in addition confirmed the presence of specific functional groups such as proteins and does have an important role as a capping and stabilizing agent in the biosynthesis of AgNPs (Al-Katib et al., 2015). Cyanobacteria could play an instrumental role as an excellent candidate for nanoparticle biosynthesis.

The article "Green Synthesis of Metallic Nanoparticles and Their Potential Applications to Treat Cancer" was retracted in 2023. Reason: plagiarized images.

### Nanoparticle Synthesis Using Algae

Algae are regarded to accumulate heavy metals and may be utilized for the biogenic synthesis of metallic nanoparticles. Dried unicellular alga *Chlorella vulgaris* could synthesize nanoparticles of diverse shapes—tetrahedral, decahedral, and icosahedral accumulated near the surface (Luangpipat et al., 2011). The extract of *Chlorella vulgaris* produced Ag nanometer scale plates at room temperature. Biosynthesis of CuFe_2_O_4_@Agnano composite from *Chlorella vulgaris* combined with ciprofloxacin confirmed promising bactericidal activity toward multidrug resistant *Staphylococcus aureus* which is a rising global risk (Kahzad and Salehzadeh, 2020). The proteins present in the algal extract perform a primary function as a stabilizing agent, reducing agent, and shape-control modifier (Xie et al., 2007). *Sargassum wightii*, a marine alga, could also synthesize extracellular Ag, Au, and Au/Ag bimetallic nanoparticles (Govindaraju et al., 2009). Rapid synthesis of extracellular Au nanoparticles with a size from 8 to 12 nm via *S. wightii* has been demonstrated by Singaravelu et al. (2007). Several other algae *Kappaphycu salvarezii* (Rajasulochana et al., 2011), *Fucus vesiculosus* (Mata et al., 2008), *Tetraselmisko chinensis* (Senapati et al., 2012), *Chondrus crispus*, and *Spirogyra insignis* (Castro et al., 2013) have been reported to synthesize Au and Ag nanoparticles (Rajasulochana et al., 2011). By using the living cells of *Euglena gracilis* microalga which have been grown under either mixotropic (exposed to light and grown in an organic carbon-enriched culture medium) or autotropic condition, the gold nanoparticles synthesized were of true yield, kinetics and colloidal stability (Dahoumane et al., 2016).

### Nanoparticle Synthesis Using Plants

The plants are considered to be more suitable compared to microbes for green synthesis of nanoparticles as they are non-pathogenic and various pathways are thoroughly researched (Figure 4). A wide spectrum of metal nanoparticles has been produced using different plants (Narayanan and Sakthivel, 2011; Iravani and Zolfaghari, 2013; Mittal et al., 2013; Das et al., 2017). These nanoparticles have unique optical, thermal, magnetic, physical, chemical, and electrical properties in comparison to their counterpart bulk material with numerous applications in numerous fields of human interest (Husseiny et al., 2007; Duran and Seabra, 2012). There are various biological entities which are used for AgNPs synthesis (Keat et al., 2015). *Jatroa curcas* extract results in the production of homogenous (10–20 nm) AgNPs from AgNO_3_ salt in 4 h (Bar et al., 2009). The leaf extracts of *Acalypha indica* have exhibited the capability to synthesize AgNPs. The size of the AgNPs obtained became extensively homogeneous and ranged from 20 to 30 nm (Krishnaraj et al., 2009). In another study, *Medicago sativa* seed exudates were used for the synthesis of AgNPs. The reduction of Ag^+^ happened almost immediately as nanoparticles had been reported within a minute of metal salt exposure and 90% of Ag^+^ was reduced at 30°C in <50 min. The resulting nanoparticles were flower-like and/or triangular and spherical with a size range of 5–108 nm and had a heterogeneous size distribution (Lukman et al., 2010). The leaf extract of *Ocimum sanctum* can also reduce Ag^+^ resulting in the AgNPs of 3–20 nm in size production The particles were spherical and stabilized by the way of a component of the leaf broth (Koduru et al., 2011). *Terminalia chebula* fruit extract has been used to promptly produce Ag nanoparticles (Jebakumar Immanuel Edison and Sethuraman, 2012). *Eucalyptus macrocarpa* leaf extract produced Ag nanoparticles of cubic shape ranging in size from 50 to 200 nm (Poinern et al., 2013); spherical gold nanoparticles of around 20 nm by *Nyctanthes arbor tristis* (night jasmine) flower extract (Das et al., 2011); leaf extract from *Coriandrum sativum* (coriander) leaf extract produce Ag and Au nanoparticles of 7–58 nm (Mittal et al., 2013). Phyllanthin extracted from the plant *Phyllanthus amarus* may be used to produce both gold and silver nanoparticles. This study is unique for the use of single constituent of a plant extract to synthesize metallic nanoparticles in comparison to different investigations wherein the whole plant was used (Kasthuri et al., 2008). The shape and size of nanoparticles produced had been affected by the concentration of phyllanthin used. Low concentrations of phyllanthin resulted in the triangular and hexagonal AuNPs formation, whereas higher concentrations produced increased spherical NPs (Kasthuri et al., 2008). Plant derived polysaccharides and phytochemicals nanoparticle (Park et al., 2011), soluble starch (Raveendran et al., 2003), cellulose (Cai et al., 2009), dextran (Ma et al., 2005), chitosan (Laudenslager et al., 2008), alginic acid (Saha et al., 2009), and hyaluronic acid (Kemp et al., 2009) may be harnessed and studied for the synthesis of silver and gold nanoparticles successfully. These compounds offer benefits of using less toxic chemical compounds and render capability to create nanocomposites with different metals. The incubation of the extract from lemon-grass plant, *Cymbopogon flexuosus*, with gold tetrachloride solution resulted in the formation of a unique type of liquid-like nanotriangles by the aggregation of spherical AuNPs, the surface of which forms a complex with the aldehydes and/or ketones present in the plant extract, contributing to the fluidity (Sangaru et al., 2004). The leaf broth of *Azadirachta indica*, forms a complex when dealing with the salts of silver, gold, and then both metallic ions concurrently produced silver, gold, and bimetallic silver-gold NPs. The rate of formation of nanoparticles became faster having attained the plateau in 2 h. The stability of NPs was attributed to the terpenoid and flavanone components of the leaf (Sangaru et al., 2004). Phytochemically reduced NiO NPs with garlic and ginger add on to the increased bactericidal activity toward multiple drug resistant *Staphylococcus aureus* which may address drug resistance issues to an extent (Haider et al., 2020).

The article "Green Synthesis of Metallic Nanoparticles and Their Potential Applications to Treat Cancer" was retracted in 2023. Reason: plagiarized images.

**Figure 4:** Green synthesis of Cds nanoparticles by bacteria.

Alloying Ag and Au has brought about the formation of bimetallic nanoparticles. Their production entails the competitive reduction between two aqueous solutions having one of a kind of metallic ion precursor used together with a plant extract. The Ag-Au nanoparticle, the core-shell structure is manufactured from Au due to its larger reduction potential, and Ag ions are reduced and form a shell with Ag coalescing on the core. Few plants have been efficiently used to synthesize Ag-Au bimetallic nanoparticles like *Azadirachta indica* (Sangaru et al., 2004), *Anacardium occidentale* (Sheny et al., 2011), *Swieteni amahagony* (Mondal et al., 2010), and cruciferous vegetable extracts (Jacob et al., 2012).

Extracts from various plants have been used to synthesize nanoparticles of copper (Cu) and copper oxide (CuO). Cu nanoparticles varying from 40 to 100 nm in size were synthesized from *Magnolia kobus* leaf extract (Lee et al., 2013) and from *Syzygium aromaticum* (Clove) (Subhankari and Nayak, 2013) showing spherical to granular shape with 40 nm of an average particle size. The Latex from the stem of *Euphorbia nivulia* (Common milk hedge) was used to synthesize an important class of Cu nanoparticles stabilized and coated through terpenoids and peptides of the latex (Valodkar et al., 2011a) and synthesis of a notably stable spherical nanoparticles of CuO was confirmed from *Sterculia urens* (Karaya gum) with a particle size of 4.8 nm (Padil and Cernik, 2013).

The synthesis of the first platinum nanoparticles was demonstrated with the help of Song et al. (2009b) *Diospyros kaki* (Persimmon) leaf extract and carboxylic acids, amines, alcohols. Ketones present in the leaf extract act as a functional group for the reduction of Pt ions. There was 90% reduction of Pt ions into nanoparticles in ~2.5 h. The possibility of an enzyme mediated process was ruled out due to the temperature of execution of the experiment (95°C) which is high enough to denature proteins. Palladium nanoparticles were synthesized using the extract of *Cinnamon zeylanicum* bark (Sathishkumar et al., 2009a,b) and *Annona squamosa* (custard apple) peel extract for the synthesis of Pd nanoparticles of size 75–85 nm (Roopan et al., 2012). Nanoparticles with a mean size of 15 nm had been synthesized from the leaf extract of soybean (*Glycine max*) (Petla et al., 2012). The extracts from commonly available *Camellia sinensis* (Tea) and *Coffe aarabica* (Coffee) have been utilized to produce nanoparticles of palladium of sizes ranging from 20 to 60 nm with faced centered cubic crystal symmetry (Petla et al., 2012). Furthermore, when an extract of *Gardenia jasminoides* (Cape jasmine) is used to synthesize nanoparticles of palladium the antioxidants (geniposide, chlorogenic acid, crocins, and crocetin) present in the extracts acts as stabilizing and reducing agents (Jia et al., 2009). Other plants like *Ocimum sanctum* leaf extract (Holy basil) (Soundarrajan et al., 2011), plant wood nanomaterials (Lin et al., 2011) and lignin from red pine (*Pinus resinosa*) were used for the synthesis of nanoparticles of platinum and palladium (Coccia et al., 2012).

The article "Green Synthesis of Metallic Nanoparticles and Their Potential Applications to Treat Cancer" was retracted in 2023. Reason: plagiarized images.

Nanoparticles of spherical size and ranging in size from 100 to 150 nm from metal oxide which includes titanium dioxide (TiO_2_) were synthesized efficaciously using numerous plant extracts *viz. Annona squamosa* peel (Roopan et al., 2012), *Cocos nucifera* coir (Roopan et al., 2013), *Nyctanthes arbor-tristis* leaf extracts (Sundrarajan and Gowri, 2011), *Psidium guajava* (Thirunavukkarasu et al., 2013), *Eclipta prostrata* (Rajakumar et al., 2011; Zahir et al., 2015), and *Catharanthus roseus* (Kanayairam et al., 2011). Spherical shaped zinc oxide (ZnO) nanoparticles were obtained using the latex of *Calotropis procera* (Singh, 2011), *Aloe vera* (Duran and Seabra, 2012), *Physalisalke kengi* (Sangeetha et al., 2011), and *Sedum alfredii* (Qu et al., 2011a,b). Biogenic Indium oxide (In_2_O_3_) spherical nanoparticles were synthesized with a variable size range from 5 to 50 nm by using leaf extracts from *Aloe vera* (*Aloe barbadensis*) (Laokula et al., 2008).

Iron (Fe) nanoparticles were synthesized by the use of green chemistry methods including the aqueous *Sorghum bicolor* bran extracts (Njagi et al., 2011) and leaf extracts of *Azadirachta indica* (Pattanayak and Nayak, 2013), *Euphorbia milii, Tridax procumbens, Tinospora cordifolia, Datura innoxia, Calotropis procera*, and *Cymbopogon citratus* (Shah et al., 2014). The latex from *Jatropha curcas* has been used to synthesize spherical Pb nanoparticles of sizes from 10 to 12.5 nm (Joglekar et al., 2011). Synthesis of metallic nanoparticles includes the use of the extracts of plant parts or whole plant extracts. Also, metallic nanoparticles may be synthesized inside living plants and a novel approach for the synthesis of PdNPs by the use of *Arabidopsis thaliana* was reportedly developed (Parker et al., 2014) by growing the plant in the usual growth medium, and medium was then replaced with potassium tetrachloropalladate (K_2_PdCl_4_) followed by the incubation for 24 h in the salt solution. PdNPs of 2–4 nm were produced as visualized by transmission electron microscope. These biologically synthesized PdNPs had been utilized in Suzuki-Miyaura coupling reactions with better catalytic activity as compared to the commercially available PdNPs (Parker et al., 2014). The Alfalfa plant seeds were grown with various concentrations of K(AuCl_4_) for 2 weeks for the formation of AuNP nanoparticles (Gardea-Torresdey et al., 2002). The time taken for the synthesis of nanoparticles via this method exceeds 2 weeks, limiting its commercial feasibility. However, if production time is reduced, it might be a great strategy for creating a cheap green method for synthesizing nanoparticles.

The article "Green Synthesis of Metallic Nanoparticles and Their Potential Applications to Treat Cancer" was retracted in 2023. Reason: plagiarized images.

### Nanoparticle Synthesis Using Viruses

Quantum dots were synthesized by using viruses over the last decade (Dameron et al., 1989; Lee et al., 2002; Mao et al., 2003) for the synthesis of nanomaterials. The outer capsid protein present on the virus offers an attractive function in the synthesis of nanoparticles by supplying a highly reactive surface interacting with metallic ions (Makarov et al., 2014). Tobacco mosaic virus (TMV) has ~2,130 capsid proteins masking its surface. These proteins act as notch attachments for the material to deposit (Royston et al., 2008; Aljabali et al., 2010; Górzny et al., 2010; Kobayashi et al., 2012) or may be used to synthesize the three-dimensional vessels for multiple applications in the pharmaceutical industry. The addition of Ag or Au salts to low concentrations of TMV prior to including plant extracts of *Nicotiana benthamiana* (Round-leaved native tobacco) or *Hordeum vulgare* (Barley) showed a decrease in the size of the synthesized nanoparticles. Additionally it accelerated their numbers as compared to those having no viral supplement (Love et al., 2014) showing relatively small free nanoparticles formation at higher TMV concentrations. TMV also served as a bio-template to form nanowires by using metallization. The unexplored potential of viruses in the manufacture of nanometer scale structures of different varieties have been reported elsewhere (Shenton et al., 1999; Merzlyak and Lee, 2006). They deliver inorganic substances such as cadmium sulfide (CdS), silicon dioxide (SiO_2_), zinc sulfide (ZnS), and iron oxide (Fe_2_O_3_). Semiconductor substances such as CdS and ZnS are utilized in electronic goods and therefore hold importance in the electronics industry.

## Factors Affecting Biological Synthesis of Metal Nanoparticles

The morphological characteristics of nanoparticles can be manipulated by means of various parameters *viz*. reaction time, reactant concentrations, pH, and temperature (Table 1). Such parameters are crucial to understand the effect of environmental factors for the synthesis of NP as they may play an important role during the optimization of metallic NPs synthesis by biological means.

The article "Green Synthesis of Metallic Nanoparticles and Their Potential Applications to Treat Cancer" was retracted in 2023. Reason: plagiarized images.

**Table 1:** Factors affecting biological synthesis of metal nanoparticles.

**S. No**	**Factors**	**Influence on biological synthesis of metal nanoparticles**	**References**
1.	pH	Size and shape of the synthesized nanoparticle	Dubey et al., 2010; Sathishkumar et al., 2010
2.	Reactant concentration	Shape of the synthesized nanoparticles	Chandran et al., 2006
3.	Reaction time	Size and shape of the synthesized nanoparticle	Tc et al., 2011
4.	Reaction temperature	Size, shape, yield and stability of the synthesized nanoparticle	Song et al., 2009a; Sathishkumar et al., 2010

### pH

The reaction medium pH plays an critical role in the formation of nanoparticles (Gardea-Torresdey et al., 1999). Size and shape of nanoparticles vary with the pH of the medium, and large sized nanoparticles are produced in acidic pH (Dubey et al., 2010; Sathishkumar et al., 2010). The rod-shaped gold nanoparticles were synthesized by using biomass of *Avena sativa* (Oat) resulting in the size range from 25 to 85 nm at pH 2 which was comparatively smaller (5–20 nm) at pH 3 and 4 (Armendariz et al., 2004). Further, accessibility of functional groups for particle nucleation in the extract was better at pH 3 or 4 as compared to the pH 2 as fewer functional groups were available prompting particle aggregation to form larger Au nanoparticles. An increased number of spherical Ag nanoparticles were synthesized in *Cinnamon zeylanicum* bark extract at higher pH (pH >5) (Kumar and Yadav, 2009). A slight increase was observed in particle size at higher pH when *Cinnamon zeylanicum* bark extract was used for the synthesis of palladium (Pd) nanoparticles, and particle size was estimated from 15 to 20 nm at pH <5, and 20–25 nm at the higher pH (Kumar and Yadav, 2009).

### Reactant Concentration

The formation of metallic nanoparticles is affected by the concentration of biomolecules present in the extract. The shape of the biosynthesized Au and Ag nanoparticles by using the sun-dried *Cinnamomum camphora* (camphor) leaf extract affected by the amount of biomass in the reaction medium (Huang et al., 2007). Exposure of the precursor chloroauric acid to growing concentrations of the extract resulted in the synthesis of spherical nanoparticles instead of triangular. A change in the ratio of spherical nanoparticles to triangular plates in the reaction medium having chloroaurate ions due to the presence of carbonyl compounds in the extract was observed when treated with varying concentrations of *Aloe vera* leaf extract (Chandran et al., 2006). Nanoparticle size can be modulated between 50 and 350 nm by using different extract concentrations (Chandran et al., 2006). Spherical, triangular, hexagonal, and decahedral shapes of AgNPs were produced by varying the concentration of *Plectranthu samboinicus* leaf extract in the reaction medium (Narayanan and Sakthivel, 2010). An increase in the variety of Ag nanoparticles was observed with increasing concentration of *Cinnamon zeylanicum* bark extract (Kumar and Yadav, 2009). The extracellular (Agnihotri et al., 2009) and intracellular synthesis (Pimprikar et al., 2009) of Au nanoparticles was affected by biomass and Au salt concentration using marine yeast, *Yarrowia lipolytica*. An increased Au salt concentration produced both nanoscale spheres and plates. In another study, a silver-tolerant yeast strain MKY3 synthesized spherical Ag nanoparticles extra-cellularly with the size ranging from 2 to 5 nm (Kowshik et al., 2003).

The article "Green Synthesis of Metallic Nanoparticles and Their Potential Applications to Treat Cancer" was retracted in 2023. Reason: plagiarized images.

### Reaction Time

The reaction time plays an important role for synthesizing nanoparticles (Ahmad, 2012). A rapid color change was observed within 2 min when *Anana scomosus* (Pineapple) extract was used for AgNPs synthesis, and aqueous AgNO_3_ solution was rapidly decreased, forming nanoparticles within 2 min. The reaction continued for up to 5 min and then there was a slight color change. The shape of synthesized nanoparticles was spherical with a mean size of 12 nm (Ahmad, 2012). *Chenopodium album* leaf extract was used for the biogenic production of Ag and Au nanoparticles. The nanoparticles were formed within 15 min of the reaction and the reaction continued over a period of 2 h and very few nanoparticles with larger size were synthesized (Dwivedi and Gopal, 2010). Change in the particle size (ranging 10–35 nm) was observed when reaction time was increased from 30 min to 4 h using *Azadirachta indica* leaf extract and AgNO_3_ (Tc et al., 2011).

### Reaction Temperature

The reaction temperature is a critical component which plays a key role in determining the shape, size, and yield of synthesized nanoparticles using plants (Song et al., 2009a; Sathishkumar et al., 2010). The peel extract of *Citrus sinensis* (sweet orange) produced particles with an average size of around 35 nm at 25°C. The average size of the nanoparticles decreased to 10 nm with the rise in the reaction temperature to 60°C (Kaviya et al., 2011). The stable Ag nanoparticles were synthesized by *Diospyros kaki* (persimmon) leaf extract at the reaction temperature varying from 25 to 95°C (Song et al., 2009b). The variation in the temperature of reaction conditions for the synthesis of Au nanoparticles using *Avena sativa* (oat) biomass ended in modifications in the shape and size of the nanoparticles produced (Armendariz et al., 2004). A higher temperature supports an increased rate of formation of Au nanoparticles. The spherical Au nanoparticles were predominantly formed at the lower temperature whereas at higher temperatures rod-like and plate-like nanoparticles were formed (Gericke and Pinches, 2006a,b). The reaction rate and particle formation rate increased with the increase in the reaction temperature. The particle conversion rate steadily increased and average particle size saw a decrease with the rise in the reaction temperature to 60°C.

The article "Green Synthesis of Metallic Nanoparticles and Their Potential Applications to Treat Cancer" was retracted in 2023. Reason: plagiarized images.

The extracellularly produced PtNPs amount was reported to be 5.66 mg l^−1^ (Riddin et al., 2006), with the variation in the temperature that affects production rates of the PtNPs. The slight change in pH from the standard inhibits the PtNPs formation (Riddin et al., 2006).

## Applications of Metallic Nanoparticles Synthesized by Green Technology

Nanoparticles have wide applications in both biomedical and physicochemical fields. They may be used for drug delivery, biosensing, bio-imaging, and biomolecular recognition (Figure 5) in bio-medical research. Such nanoparticles are integrated in various materials of everyday use which includes cosmetics, toothpaste, deodorants, water purification systems, and humidifiers due to their anti-microbial properties (Baker et al., 2005). They have an important role to play in agriculture technology such as detection and abatement of plant diseases and minimizing nutrient leaching to increase the crop yield. They are also used in solar and oxide batteries for energy storage.

**Figure 5:** Application of Green synthesis of metallic nanoparticles.

### Gold and Silver Nanoparticles

The variation in shape, size, and surface properties of Au nanoparticles (Wang et al., 2005; Ghosh and Pal, 2007; Cai et al., 2008; Alexandridis, 2011; Shivaji et al., 2014) makes them very beneficial for their potential applications within the area of biosensors (Chan and Nie, 1998; Kreibig and Vollmer, 2013), hyperthermia therapy (Huang et al., 2006), delivery systems for therapeutic drugs and genetic materials (Paciotti et al., 2004), as well as anti-bacterial drugs (Sondi and Salopek-Sondi, 2004; Hsiao et al., 2006). Gold nanoparticles from *Sesbaniadrum mondii* (rattlebush) have shown the catalytic activity that may be beneficial in the reduction of aromatic nitro compounds in waste decontamination.

The rise in antibiotic resistance among pathogenic bacteria has highlighted the antibacterial properties of nanoparticles and their ability to be used as new medical tools. The antimicrobial activity of Ag is widely known and is used in multiple medical preparations against pathogens (Sondi and Salopek-Sondi, 2004; Kumar and Yadav, 2009; Sotiriou and Pratsinis, 2011). The anti-bacterial properties of AbNPs have allowed for their extensive use in food storage, the health industry, textile coatings and several environmental applications. Silver nanoparticles synthesized by the use of *Tridax procumbens* (tridax daisy) extract have robust antibacterial activity toward *Escherichia coli, Shigella dysenteriae*, and *Vibrio cholera* (Dhanalakshmi and Rajendran, 2012). Silver nanoparticles obtained by using *Pinusthun bergii* (Japaneseblack pine) cone extracts exhibit antibacterial activity against diverse Gram-negative and Gram-positive agricultural pathogens (Velmurugan et al., 2012), and the antifungal effect of Ag nanoparticles has been confirmed (Vivek et al., 2011). Their utility as antifungal agents is found to be safer as compared to the conventional fungicides (Park et al., 2011). Ag nanoparticles interact closely with the bacterial cell membrane due to their high surface area to volume ratio as well as size (Chen and Schluesener, 2008). Recent antimicrobial studies of Ag nanoparticles have shown that they can cause significant membrane damage and DNA toxicity via bio-sorption and cellular uptake (Brayner et al., 2006; Simon-Deckers et al., 2009). AgNPs are already in-use as antimicrobial agents in many commercially available medical and consumer goods. Despite decades of its use, it is important to note that the evidence of the silver toxicity is not yet fully explored. Their applications have been discovered both in the field of medicine and home remedies. Silver sulfadiazine creams are often used to prevent burn site infection and some companies have also built silver into their washing machines. Presently, silver seems be a part of many consumer products such as computer keyboards, acne creams, and clothing (e.g., socks and athletic wear) that protects the wearer from emitting body odor further to deodorizing sprays. A range of organizations that offer accreditation like US-FDA, US-EPA, Korea's Testing, SIAA of Japan and Research Institute for Chemical Industry and FITI Testing and Research Institute have approved products containing silver nanoparticles (Veeraputhiran, 2013). The silver nanoparticles also display an anti-tumorigenic ability due to their cytotoxic activity against various tumor cells. The growth and survival of HeLa cells were inhibited by the silver nanoparticles synthesized from *Iresine herbstii* (Herbst's bloodleaf). AgNPs produced by latex extracts of *Euphorbia nivulia* (leafy milk hedge) exhibited toxicity toward the human lung cancer cells (A549) (Valodkar et al., 2011b). *Nerium oleander* (oleander) extracted silver nanoparticle displayed robust larvicidal activity against malaria vector larvae (Suganya et al., 2013), as optical sensors that form small molecule adsorbates (McFarland and Duyne, 2003), as selective and sensitive nanoscale affinity biosensors to investigate the transport across the membrane of living microbial cells (*P. aeruginosa*) in real time (Xu et al., 2004). Silver nanoparticles and their composites demonstrate better catalytic activities in dye reduction and their elimination (Kundu et al., 2002; Mallick et al., 2006).

The article "Green Synthesis of Metallic Nanoparticles and Their Potential Applications to Treat Cancer" was retracted in 2023. Reason: plagiarized images.

### Copper and Copper Oxide Nanoparticles

The nanoparticles of CuO display anti-oxidant, anti-bacterial, and antimicrobial activity against common pathogenic strains such as *Escherichia coli* and *Staphylococcus aureus* and are shown to have tremendous application potential (Heinlaan et al., 2008; Das et al., 2012; Padil and Cernik, 2013). Cu nanoparticles have antibacterial potential against common pathogenic bacteria *Escherichia coli* (Lee et al., 2011). They have functional decontaminating properties against several infectious micro-organisms with the potential to be used as bactericidal material (Akhavan and Ghaderi, 2010; Hassan et al., 2012; Subhankari and Nayak, 2013). The Cu nanoparticles synthesized by stem latex of *Euphorbia nivulia* were seen toxic to human lung cancer cells (A549) (Valodkar et al., 2011c) surfacing the their potential application in the field of cancer therapy.

### Palladium and Platinum Nanoparticles

The catalytic activity of platinum nanoparticles extracted from *Ocimum sanctum* (Holy basil) for the electrolysis of water to produce hydrogen fuel elements has been studied (Soundarrajan et al., 2011). A few Pt nanoparticle based catalysts show elevated activity for the electro-oxidation of formic acid used for the cleaning of surroundings (Waszczuk et al., 2002).

### Titanium Dioxide and Zinc Oxide Nanoparticles

TiO_2_ suspensions have been explored successfully for both adulticidal and larvicidal properties against *Hippobosca maculate* (hematophagous fly) and *Bovicolaovis* (sheep louse) (Kanayairam et al., 2011). TiO_2_ nanoparticles synthesized from the extract of *Psidium guajava* confirmed the effective antibacterial activity against *Aeromona shydrophila, Escherichia coli, Proteus mirabilis, Pseudomonas aeruginosa*, and *Staphylococcus aureus*, pathogens with strong antioxidant behaviors (Heinlaan et al., 2008; Thirunavukkarasu et al., 2013). TiO_2_ oxide nanoparticles have shown applications in the biomedical industry, disinfection of waste water, and beauty products. ZnO nanoparticles additionally possess antibacterial activity that was used in waste water treatments and food packaging (Espitia et al., 2012). Biogenic ZnO nanoparticles can be used as a drug delivery vehicle for doxorubicin (Vimala et al., 2013). The nanoparticles of magnetite were used in biomedical applications such as magnetic resonance imaging (Sun and Zeng, 2002; You et al., 2013) and oscillation damping and position sensing (Thapa et al., 2004). Furthermore, afore-mentioned NPs have many non-medical applications that include magnetic recording devices.

The article "Green Synthesis of Metallic Nanoparticles and Their Potential Applications to Treat Cancer" was retracted in 2023. Reason: plagiarized images.

## Conclusion and Future Perspective

Green synthesis technology presents a clean, non-toxic and eco-friendly technique for the synthesis of metallic nanoparticles and is of enormous interest due to economic prospects and feasibility. However, protocols need to be modified further for making these methods cost-effective and comparable with traditional methods for the large-scale production of nanoparticles. Improvement of reliable and eco-friendly processes for the synthesis of metallic nanoparticles is a significant step in the field of applied nanotechnology. Further, most of these strategies are still under the developmental stage and challenges need to be taken care of. These encompass stability and aggregation of nanoparticles, managing the crystal growth, morphology and size. The separation and purification of nanoparticles is another vital parameter which needs to be explored further. Metal nanoparticles produced by the plants and/or plant extracts are more stable as compared to those produced through different organisms. Genetically modified organisms (GMO) have tremendous capability to optimize for generating a greater quantity of proteins, enzymes, and biomolecules required for the biosynthesis and stabilization of nanoparticles. We believe genetic change to enhance the metal tolerance and accumulation capacity is the future approach to enhance the production of metal nanoparticles by adopting the “green synthesis” approach.

## Author Contributions

DZ and G-wZ conceived the idea, designed study, executed, and wrote the paper. X-lM, YG, HH, and G-wZ helped during formulation of this article and approved. All authors contributed to the article and approved the submitted version.

## Conflict of Interest

The authors declare that the research was conducted in the absence of any commercial or financial relationships that could be construed as a potential conflict of interest.
